# Breast cancer-released exosomes trigger cancer-associated cachexia to promote tumor progression

This article has been retracted.

**DOI:** 10.1080/21623945.2018.1551688

**Published:** 2018-12-11

**Authors:** Qi Wu, Si Sun, Zhiyu Li, Qian Yang, Bei Li, Shan Zhu, Lijun Wang, Juan Wu, Jingping Yuan, Changhua Wang, Juanjuan Li, Shengrong Sun

**Affiliations:** a Department of Breast and Thyroid Surgery, Renmin Hospital of Wuhan University, Wuhan, Hubei, P. R. China; b Department of Clinical Laboratory, Renmin Hospital of Wuhan University, Wuhan, Hubei, P. R. China; c Department of Pathology, Renmin Hospital of Wuhan University, Wuhan, Hubei, P. R. China; d Department of Pathophysiology, Wuhan University School of Basic Medical Sciences, Wuhan, Hubei Province, P. R. China

**Keywords:** Breast cancer, exosomes, cachexia, tumour progression

## Abstract

Cancer-secreted exosomes are emerging mediators of cancer-associated cachexia. Here, we show that miR-155 secreted by breast cancer cells is a potent role on the catabolism of adipocytes and muscle cells through targeting the PPARγ. After cocultivated with mature adipocytes or C2C12, tumour cells exhibit an aggressive phenotype via inducing epithelial-mesenchymal transition while breast cancer-derived exosomes increased catabolism and release the metabolites in adipocytes and muscle cells. In adipocytes, cancer cell-secreted miR-155 promotes beige/brown differentiation and remodel metabolism in resident adipocytes by downregulating the PPARγ expression, but does not significantly affect biological conversion in C2C12. Likewise, propranolol ameliorates tumour exosomes-associated cachectic wasting through upregulating the PPARγ expression. In summary, we have demonstrated that the transfer of miR-155 from exosomes acts as an oncogenic signal reprograming systemic energy metabolism and leading to cancer-associated cachexia in breast cancer.

## Introduction

Cachexia is a devastating syndrome characterized by loss of skeletal muscle mass and fat mass that accompanies many chronic pro-inflammatory diseases including cancer.^1^ Importantly, cachexia occurs in more than 50% of cancer patients, especially in pancreatic and advanced breast cancer.^2,3^ Cancer-associated cachexia (CAC), an important adverse prognostic factor, not only increases patient morbidity and mortality but also reduces the efficacy of treatment.^4,5^ However, there is no explicit mechanism about tumuor-derived factors that simulate catabolism in muscle and adipose tissue considered the main characteristics of cachexia progression. Consequently, exploring the pro-cachectic factors and developing interventions is considered the key event for preventing or reversing cachexia.

The mechanism about cancer-triggered weight loss is highly complex. Loss of skeletal muscle in CAC derives from a decrease in protein synthesis and an activated protein-degradation pathways that degrades specific regulatory proteins, mitochondria and other cellular components.^1^ Emerging evidence indicates that elevations of systemic inflammation have been observed in cachectic patients and chronic inflammation such as interleukin-6 increase UCP1 expression in white adipose tissue (WAT), and reduce inflammation or β-adrenergic blockade rescues the severity of cachexia.^6^ Likewise, cytokines such as IL-1α/β and TNFα mediate cachectic states, resulting from augmenting energy expenditure in muscle cells through p38/PGC-1 axis.^7^ These data suggest that systemic inflammation is pivotal to the catabolism activation during cancer cachexia. However, the precise mechanism that cancer contributes to the catabolism in muscle and fat in discrete locations is poorly defined.

Exosomes, as small extracellular vesicles (30–100 nm), originate from the endosomal compartment of virtually all cells.^8^ Moreover, exosome content consists of mRNA, ncRNA, transcription factors, proteins, and lipids, and exosomes have been implicated in cell communication and the modulation of cell biology by trafficking these materials into target recipient cells.^9^ It is evident that tumor exosomal Hsp70 and Hsp90 as key cachexins play a primary role in muscle wasting.^10^ In addition, exosomal miRNA profiles parallel those of the originating tumor cells.^11^ Although exosomes derived from tumor cells are related to muscle cell death in cancer cachexia,^12^ their potential role in the neoplastic-transformed cachexia has not been elucidated. Thus, we hypothesize that the underlying mechanism involves the delivery of special onco-miRNAs from breast cells to adipocytes and skeletal muscle via exosomes resulting in CAC.

Here, we report that adipocytes and muscle cells increase energy expenditure and release metabolites, such as lactate, pyruvate and free fatty acids (FFAs), upon receipt of tumor-derived exosomes to promote tumor metastasis. Our data show that specific miRNAs in these exosomes are associated with the pro-tumorigenic process. Our work suggests that tumor-derived exosomes are novel factors that promote tumor progression by increasing catabolism in muscle cells and adipocytes, promising therapeutic targets for conquering CAC.

## Results

### Breast cancer-derived exosomes rewrite metabolic characteristics in adipocytes

Breast cancer cells invade regions of adipocytes in the tumor microenvironment.^13^ Therefore, we assessed the possibility that stromal adipocytes contribute to the increased expression of catabolite transporters detected in samples from patients with breast cancer and affirmed the significance of these biomarkers in breast cancer malignancy. For these purposes, we initially detected the expression of fatty acid transport protein-1 (FATP1) and CD36 (also called fatty acid translocase) in a cohort of 108 breast cancer specimens using immunohistochemistry (IHC). High expression of CD36 and FATP1 was detected in most breast cancer tissues with predominant localization proximal to adipose tissue (Figure 1A). Furthermore, Kaplan-Meier analysis revealed that patients with FATP1 or CD36 overexpression in breast cancer tissue had a poorer survival time than patients with those protein underexpression (Figure 1B, P < 0.01 and P = 0.019, log-rank test). These findings suggest that overexpression of CD36 or FATP1 in malignant tissue may serve as important clinical biomarkers for the poor prognosis of breast cancer patients.

**Figure 1.** Breast cancer-derived exosomes reshape metabolic characteristics in adipocytes and metabolite biomarkers in breast cancer are linked to a poor prognosis. (A) Representative immunohistochemistry staining of CD36 and FATP1. The pictures also show positive staining for FATP1 and CD36 in breast cancer tissues located near stromal adipocytes. (B) Kaplan-Meier survival analysis of patients with biomarker-positive and biomarker-negative IHC staining. (C) Mature adipocytes after treated were stained with red oil. The adipocytes in the CytoD group were treated with cytochalasin D (final concentration, 2 μg/ml) and 50 μg of exosomes purified from cancer-associated conditioned medium (CA-CM) (enlarged 100X). (D) The levels of secreted metabolites (glycerol and free fatty acids) enriched in media were determined by colorimetric assay. AD: adipocytes. (E) Raw data for the oxygen consumption rate (OCR) and extracellular acidification rate (ECAR) as determined by the Seahorse XF24 analyzer. The ECAR was evaluated after the addition of 10 mM glucose to adipocytes in the presence or absence of exosomes. The OCR was measured in the presence of palmitate as described in the Methods. (F) Adipocytes were cocultivated in the presence or absence of exosomes. After 3 days, proteins were extracted for western blot analysis of the expression of the indicated proteins. The numbers represent the relatively quantitative results compared to the control group. Data are presented as the mean ± S.D. of at least three independent experiments. * P < 0.05 versus control values.

Adipocytes promote tumor growth and invasion in vitro and in vivo,^14–16^ but the mechanism by which they contribute to cancer metastasis remains unclear. Mature adipocytes cocultivated with breast cancer cells displayed a dramatic reduction in lipid droplet size and number (Figure 1C). Moreover, our results demonstrated that tumor-surrounding adipocytes appeared to be undergoing a lipolytic process. Glycerol and FFAs, the products of TG hydrolysis, were released by adipocytes incubated with both MDA-MB-231 and MCF-7 cells (Figure 1D). To confirm if this change in adipocytes was indeed due to exosome uptake, we added cytochalasin D (CytoD), an endocytosis inhibitor, to mature 3T3-L1 culture media supplemented with exosomes purified from CA-CM. Notably, CytoD partially inhibited lipolysis and decreased in metabolites in CA-CM (Figure 1C, D). In parallel, the ECAR in response to glucose was increased after cocultured with exosomes, demonstrating that anaerobic glycolysis was already maximal in cocultivated adipocytes in the presence of glucose. We then investigated the OCR in conditions that favor FAO (Krebs medium with palmitate, carnitine, and restricted glucose). In these conditions, the OCR was decreased in cocultivated cells compared with non-cocultivated cells (Figure 1E). Therefore, the results indicate that breast cancer cell-derived exosomes remodel metabolism in adipocytes.

Previous studies have shown that mammary fat in the tumor microenvironment overexpresses UCP1 and exhibits a catabolic stroma.^6^ Thus, we next evaluated if adipocytes undergo beige/brown differentiation, as assessed by the upregulation of UCP1 and the induction of a catabolic stromal phenotype. First, we assessed the levels of UCP1, Figure 1F shows that adipocytes cocultivated with tumor exosomes harbored increased UCP1 levels compared with adipocytes cultivated alone and CytoD partially reduced UCP1 levels in cocultured adipocytes. We next evaluated the expression levels of P-P38, P-ERK1/2, PPARγ and P-PPARγ as primary markers of catabolic modulation. Figure 1F shows that P-P38 was upregulated but P-ERK1/2 was downregulated in adipocytes incubated with the exosomes from both MDA-MB-231 and MCF-7 cells relative to normal adipocytes. The protein level of PPARγ and P-PPARγ, which is involved in lipid accumulation, was dramatically reduced in cocultivated adipocytes (Figure 1F). Taken together, the findings indicate that cancer cells induce the beige/brown differentiation of adipocytes and promote adipocyte catabolism.

### Breast cancer-secreted exosomes remodeled metabolic process in skeletal muscle cells

Tumor exosomes were identified to induce muscle catabolism in vitro and in vivo,^10,12^ but the mechanism remains unclear. Mature muscle cells differentiated from murine C2C12 myoblasts cocultivated with the exosomes from breast cancer cells displayed a plenty of cell death within 24 h (data not shown), a spot of the rest was observed to stimulate myosin heavy chain 1 (MYH1) loss and myotube atrophy (Figure 2A). Moreover, our results demonstrated that tumour-induced muscle cells appeared to be undergoing a catabolic process. Pyruvate and lactate accumulated in conditioned medium (Figure 2B). To confirm if this change in muscle cells was indeed due to exosome uptake, we added cytochalasin D (CytoD) to mature C2C12 culture media supplemented with exosomes purified from conditioned medium. Notably, CytoD partially inhibited the increase in metabolites in medium (Figure 2B). As shown in Figure 2C, the ECAR in response to glucose was increased after treated by exosomes, demonstrating that anaerobic glycolysis was already maximal in cocultivated C2C12 in the presence of glucose. We then investigated the OCR in conditions that favor FAO (Krebs medium with palmitate, carnitine, and restricted glucose). In these conditions, the OCR was decreased in cocultivated cells compared with non-cocultivated cells (Figure 2C). To explore the underlying mechanism, we next evaluated if C2C12 occurs energy expenditure, as assessed by the upregulation of UCP3 and the induction of a catabolic phenotype. First, Figure 2D shows that C2C12 cocultivated with tumor exosomes harbored increased UCP3 compared with muscle cells cultivated alone and CytoD could inhibit the expressed level. We next found elevated P-P38 expression but significantly lower P-ERK1/2 expression in C2C12 cocultivated with tumoral exosomes than in muscle cells alone (Figure 2D). We next evaluated the expression levels of P-PPARγ and PPARγ as primary markers of catabolic modulation, indicating that P-PPARγ and PPARγ were dramatically downregulated in C2C12 incubated with the exosomes from both MDA-MB-231 and MCF-7 cells relative to normal muscle cells and this finding was supported by the use of CytoD that partially reversed those protein levels. Taken together, the findings indicate that cancer cells induce anomalous conversion of muscle cells and promote catabolism of muscle cells.

**Figure 2.** Skeletal muscle cells undergo extensive metabolism changes after treated breast cancer-secreted exosomes. (A) Immunofluorescence staining for myosin heavy chain 1 (MYH1) after treatment 24 h. Scale bars represent 50 μm. The C2C12 in the CytoD group were treated with cytochalasin D (final concentration, 2 μg/ml) and 50 μg of exosomes purified from cancer-associated conditioned medium (CA-CM). (B) The levels of secreted metabolites (pyruvate and lactate) enriched in media were determined by colorimetric assay. (C) Raw data for the oxygen consumption rate (OCR) and extracellular acidification rate (ECAR) as determined by the Seahorse XF24 analyzer. The ECAR was evaluated after the addition of 10 mM glucose to C2C12 in the presence or absence of exosomes. The OCR was measured in the presence of palmitate as described in the Methods. (D) C2C12 were cocultivated in the presence or absence of exosomes. After 24 h, proteins were extracted for western blot analysis of the expression of the indicated proteins. The numbers represent the relatively quantitative results compared to the control group. Data are presented as the mean ± S.D. of at least three independent experiments. * P < 0.05 versus control values, # P < 0.05 versus control values as positive group.

### Tumour cells cocultivated with mature adipocytes or skeletal muscle cells exhibit an aggressive phenotype

We questioned whether adipocytes or muscle cells stimulate the invasive ability of breast cancer cells by inducing epithelial-mesenchymal transition (EMT) by coculture. As shown in Figure 3A, the migration abilities of both MDA-MB-231 and MCF-7 cells in a wound healing assay were significantly improved with conditioned medium compared with controls at 24 hours (Figure 3A). Moreover, an invasion assay also demonstrated a profound increase in the number of invasive cells in the presence of conditioned medium (Figure 3B). Meanwhile, CytoD could reverse cancer-stimulated migration capacity and invasiveness. Ultimately, the downregulation of E-cadherin, an EMT-related marker, was observed in the presence of mature 3T3-L1 cells or mature C2C12 relative to the absence of those (Figure 3C). Hence, our results show that adipocytes or muscle cells promote the invasiveness of breast tumor cell in vitro.

**Figure 3.** Tumor cells exhibit increased invasion capacities upon coculture with adipocytes or muscle cells. Cancer-associated conditioned medium (CA-CM) was collected from adipocytes cultivated with MCF-7 or MDA-MB-231 cells for 3 days or C2C12 cultivated with MCF-7 or MDA-MB-231 cells for 1 days, and adipocyte or C2C12-conditioned medium (AD-CM) were collected from cells cultivated alone as controls. All media contained 10% FBS. Wound healing assays were used to examine the effects of CA-CM from adipocytes (A) and C2C12 (B) on cell motility (Scale bar: 10 μm). Tumour cells were cultivated in control medium or CA-CM from adipocytes (C) and C2C12 (D). After 24 hours, the number of cells penetrating the membrane in Transwell invasion assays was analyzed. (E) E-cadherin protein expression was analyzed by western blot in extracts from tumor cells cocultivated in the presence or absence of adipocytes (3 days) or C2C12 (1 day). The numbers represent the relatively quantitative results compared to the control group. The bars represent the mean ± SD of triplicate datapoints (n = 3). * P < 0.05 versus control values, # P < 0.05 versus control values as positive group.

### Cocultivated breast cancer cells show altered exosomal miRNA profiles

Exosomes were isolated from conditioned medium derived from MDA-MB-231 cells cocultivated with mature adipocytes for 3 days. The purified particles displayed typical exosome morphology and size and contained CD36, TSG101 and CD81 (Figure 4A–C), which was consistent with previous reports on exosomes.^9^ To observe exosome uptake by adipocytes, breast cancer-secreted exosomes were labeled with red fluorescence. After being treated with exosomes for 4 hours, mature 3T3-L1 cells were densely packed with exosomes (Figure 4D), indicating rapid cellular uptake of exosomes by adipocytes.

**Figure 4.** Breast cancer cells cocultured with adipocytes show altered exosomal miRNA expression profiles. (A) Exosomes originating from CA-CM viewed by electron microscopy (scale bar, 200 nm). (B) Exosomes from CA-CM were analyzed by western blot. (C) NanoSight analysis of exosomes derived from CA-CM. (D) Labelled tumor cell-secreted exosomes (red) were incubated with the indicated adipocytes. (E) miRNA microarray analysis of purified exosomes from control groups and CA-CM. The heatmap shows the top 40 differentially expressed miRNAs among different groups. (F) MDA-MB-231 were cocultivated in the presence or absence of adipocytes. After 3 days, exosomal miRNAs were further verified by qPCR. And RNA was extracted from the adipocytes and subjected to qPCR analysis with primers specific to mature miRNA. Data are presented as the mean ± S.D. of at least three independent experiments. * P < 0.05 versus control values.

Many studies have confirmed that miRNAs can be transported between tumor cells and stromal cells, such as fibroblasts, macrophages and endothelial cells.^17,18^ Therefore, we attempted to identify the miRNA content that was transferred from breast cancer cells to adipocytes. miRNA microarrays were utilized to analyze exosomes in conditioned medium, and intracellular and exosomal miRNAs from MCF-10A and MDA-MB-231 cells were extracted from a GEO dataset (GSE50429) as a control. The exosomal miRNA sequencing analysis revealed distinct differences between the exo-miRNA profiles derived from normal MDA-MB-231 cells and conditioned medium. The top 40 differentially expressed miRNAs are shown in Figure 4E. Due to some miRNAs such as miR-126, miR-144 and miR-21 have been validated in previous researches, we selected miR-155 for further investigation. Among the most highly expressed miRNAs in the exosome microRNA profile, miR-155 showed much higher expression levels in exosomes of conditioned medium than in control exosomes, and this finding was confirmed by RT-PCR (Figure 4F). In addition, the expression of mature miR-155 was significantly increased in adipocytes cultivated with MDA-MB-231 cells compared to adipocytes cultured alone, but pre-miRNA levels were not detected in either group (Figure 4F). Together, these data support that breast cancer cells cocultivated with adipocytes show increased expression of miR-155 expression, which are subsequently released via the exosome pathway.

### Exosomal miR-155 from breast cancer cells mediates the adipocyte metabolism

Then, we sought to determine the mechanism by which exomiR-155 dysregulation leads to the metabolic remodeling of adipocytes. To address this question, we attempted to identify target genes and pathways modulated by miR-155. Previous studies demonstrated that miR-155, acting as a negative regulator, directly binds to the 3ʹ-UTR of PPARγ and inhibits the expression^19^; thus, PPARγ was assumed to be a particularly relevant miR-155 target gene.

One potential conserved seed site was identified by TargetScan, PicTar and miRBase upon alignment of miR-155 with the human PPARγ 3ʹUTR sequence (Figure 5A). We next established a luciferase reporter containing the human PPARγ 3ʹUTR and cotransfected it with pre-miR-155 mimic or pre-miRNA-control into HEK 293 cells. We also used a PPARγ 3ʹUTR construct harboring a mutation in the predicted miR-155 site as a control. The results showed a significant decrease in normalized luciferase activity of the wild-type construct in the presence of human pre-miR-155 relative to control, while this luciferase activity was rescued by the mutated 3ʹUTR of human PPARγ (Figure 5B). This finding demonstrates that PPARγ is indeed a direct target of miR-155.

**Figure 5.** ExomiR-155 mediates the adipocyte metabolism by downregulating PPARγ. The adipocytes in 50 μg of exosomes purified from cancer-associated conditioned medium (CA-CM). (A) The predicted miR-155 binding site in the 3ʹUTR of the PPARγ gene from TargetScan. (B) The GV272 vector containing the 3ʹUTR of the target gene harboring wild-type (wt) or mutated (mt) miRNA binding sites was transfected into HEK 293T cells stably expressing miRNA or empty vector (as a control). Luciferase activity was analyzed at 48 hours post-transfection, and the ratio of firefly luciferase activity to Renilla luciferase activity is shown. (C) Breast cancer cells were transfected with the control vector or miR-155 inhibitor, mature adipocytes were transfected with miR-155 mimic as the positive control and the control vector was applied as the negative control. Mature adipocytes cultured in the presence or absence of tumor exosomes for 3 days were stained with red oil (D), and Western blot analysis of related protein expression in different groups. The numbers represent the relatively quantitative results compared to the control group. Data are presented as the mean ± S.D. of at least three independent experiments. * P < 0.05 versus control values.

As miR-155 downregulates PPARγ level, we investigated whether the decreased PPARγ levels in cocultured adipocytes are associated with an increase in exomiR-155 expression. We transfected pre-miR-155 into mature 3T3-L1 cells as the positive control group and treated mature 3T3-L1 cells with exosomes from conditioned medium and miR-155 knockdown in cultured breast cancer cells. It was evident that mature adipocytes in the presence of breast cancer cells and overexpressing miR-155 displayed a decrease in lipid droplet compared to the positive control, and miR-155 knockdown in cultured breast cancer cells rescued lipid droplet accumulation (Figure 5C). As shown in a previous study, the inhibition of PPARγ phosphorylation at S273 induces UCP1 overexpression in adipocytes.^20^ As shown by our results, total and phosphorylated PPARγ levels significantly decreased in adipocytes incubated with breast cancer cells and adipocytes overexpressing miR-155, while miR-155 knockdown in cultured breast cancer cells rescued the reduced levels (Figure 5D). These consistent results were confirmed by UCP1 expression (Figure 5D). Further, the level of phosphorylated P38 was notably elevated but the P-ERK1/2 level was markedly reduced in adipocytes incubated with breast cancer cells and in adipocytes overexpressing miR-155, whereas these levels were restored upon miR-155 inhibition in cultivated breast cancer cells (Figure 5D). In contrast, miR-155 did not significantly influence glycolysis in C2C12 (data not shown), speculating that other miRNAs maybe determine glycolysis changes in C2C12 like miR-105.^21^ However, we did not further explore. Altogether, these experiments demonstrate that miR-155 derived from breast cancer cell exosomes mediates the energy metabolism of adipocytes thorough the downregulation of the PPARγ.

### Activated PPARγ ameliorates tumor exosomes-associated cachectic wasting

Previous studies have demonstrated that adrenergic control of thermogenesis in diverse tissue is mediated mainly by the PPARγ activator,^22^ and propranolol, which was identified as extensive β-adrenergic receptors blockade and activated the PPARγ expression, partially reverses cancer cell–induced lipolytic activation.^14^ To assess whether propranolol could prevent tumor exosomes-induced cachectic wasting, we performed studies in adipocytes differentiation and C2C12 myotubes treated tumor exosomes, showing that propranolol could rescue the tumor exosomes-induced the reduction of lipid drop in adipocytes and MYH1 loss in C2C12 (Figure 6A, C). As shown in Figure 6B, P-PPARγ and PPARγ were suppressed by exosomes originated from tumor cells, while treating cells with propranolol restored P-PPARγ and PPARγ expression. Moreover, increased P-P38 expression but reduced P-ERK1/2 level were observed in adipocytes cultured with tumor exosomes, while propranolol could reverse the protein expression (Figure 6B, D). The consistent results were observed in UCP1 and UCP3 expression (Figure 6B, D). In summary, our results indicate that propranolol prevents tumor exosomes-induced catabolic activation in adipocytes and muscle cells.

**Figure 6.** Propranolol ameliorates tumor exosomes-associated cachectic wasting in vitro. The adipocytes or C2C12 in 50 μg of exosomes purified from cancer-associated conditioned medium (CA-CM) and/or Propranolol (PRO, 10 μM). (A) Mature adipocytes in the presence or absence of exosomes and/or Propranolol were stained with red oil (enlarged 100X). (B) Adipocytes were cocultivated in the presence or absence of exosomes and/or Propranolol. After 3 days, proteins were extracted for western blot analysis of the expression of the indicated proteins. (C) Immunofluorescence staining for myosin heavy chain 1 (MYH1) after treatment 24 h. Scale bars represent 50 μm. (D) After C2C12 cells were treated for 1 days, and Western blot analysis of related protein expression in different groups. The numbers represent the relatively quantitative results compared to the control group. Data are presented as the mean ± S.D. of at least three independent experiments. * P < 0.05 versus control values, # P < 0.05 versus control values as positive group.

### Discussion

Originally cachexia is conceived as a state of ‘‘autocannibalism,’’ in which tumors are considered metabolic parasites, seizing metabolites from the resources of the depleted organism, cachexia is now described as an inflammatory and neuroendocrine response. Here, we demonstrate that high levels of exosomal miRNAs constitutively released is an essential characteristic of CAC, and that tumor cell-secreted exosomes stimulate catabolism in adipocytes and muscle cells resulting in lipolysis and muscle loss. In addition, tumor-derived exo-miR-155 induces energy expenditure of adipocytes through targeting PPARγ. Further, we show that propranolol prevents tumor exosomes-induced fat lipolysis and muscle atrophy in vitro (Figure 7). These results depict tumor-released exosomes as key cachexins responsible for CAC.

**Figure 7.** Working model for how breast-cancer-secreted exosomes reprogram metabolism in adipocytes and muscle cells to promote tumor progression. Breast cancer cells could secrete exosomes containing some special miRNAs including miR-155, which induce mitochondrial uncoupling and promote catabolism in adipocytes and muscle cells. High-energy metabolites released from adipocytes and muscle cells can be transported into breast cancer cells to remodel tumor metabolism and promote tumor progression. Moreover, propranolol ameliorates tumor exosomes-associated cachectic wasting through upregulating the PPARγ expression.

The preliminary step of this symbiosis is the ability of tumor cells to induce beige/brown differentiation and the lipolytic process in adipocytes. Our results showed that adipocytes presented beige/brown characteristics and an activated phenotype. As shown in previous studies, cancer-associated fibroblasts (CAFs) overexpress UCP1 to significantly promote breast cancer growth via the production of high-energy mitochondrial fuels containing lactate, pyruvate and FFAs,^23^ and multiple key enzymes in the catabolic process are increased in tumor-surrounding adipocytes, which is consistent with our results.^24^ Moreover, beige/brown adipose markers are enriched in host cells to stimulate tumor growth,^25^ and autophagy is activated by upregulating UCP1 levels, inducing lipolysis and generating metabolites.^23,26^ However, it indicated that energy wasting in cancer cachexia was not dependent on UCP1, but relied on AMP-activated protein kinase (AMPK) inactivation and degradation to promote energy-costly lipid.^27^ In addition, AMPK phosphorylates ATGL at S406 and HSL at S565 to stimulate lipolysis,^28^ acutely regulates glycolysis by phosphorylating PFKFB3 (6-phosphofructo-2-kinase/fructose-2,6-biphosphatase 3),^29^ and induces ketogenesis through the activation of PPARα.^30^ Thus, these data demonstrate that upon crosstalk with breast cancer cells, adipocytes increase catabolism and transfer energy to sustain tumor cell invasion.

Skeletal muscle cells in models under CAC have previously been shown to exert significant changes in proliferation, metabolism, and differentiation.^31–34^ Previous finding presented that an upregulation of UCP3 expression accompanied by a downregulation of PGC-1β expression provide evidence of mitochondrial uncoupling in cancer cachexia^35^. Also our results corroborate the previous study in part. In addition, multiple cytokines such as TNFα, IL-6 or IL-1 were observed to trigger weight loss of skeletal muscle in CAC.^36,37^ The observation had also shown that cytokines activated the transcriptional PPAR gamma coactivator-1 (PGC-1) through phosphorylation by p38 kinase, resulting in increasing the expression of genes linked to mitochondrial uncoupling and energy expenditure like UCP3.^7^ Therefore, anti-cytokine treatment prevented the depletion of muscle mass and significantly reduced the activity of muscle proteolytic systems.^38,39^ Taken together, the data indicate that the systemic inflammation in CAC was responsible for skeletal muscle atrophy through reinforcing mitochondrial uncoupling.

Exosomes play a pivotal role in the metabolic symbiosis between stromal cells and multiple types of cancer cell.^40^ Recent results indicate that exosomes derived from adipocytes carry proteins that promote cancer cell migration and invasion by increasing FAO,^40^ while exosomes secreted by pancreatic cancer cells induce lipolysis in subcutaneous adipose tissue,^41^ suggesting that exosomes have bidirectional effects on the interactions between cancer cells and host cells. Our study revealed the exomiR-155, acting as an important communicator between tumor cells and adipocytes, promoted the beige/brown differentiation and the metabolic reprogramming in adipocytes. miR-155 serves as an tumor promotor in multiple cancers,^42–44^ and mediates treatment resistance.^45^ Likewise, miR-155 was a key regulator of glucose metabolism in cancer through PIK3R1-PDK/AKT-FOXO3a-cMYC axis.^42^ Current study provided strong evidence that an enrichment in exomiR-155 from cancer stem cells transfer to breast cancer cells, resulting in increasing chemoresistance.^46^ Moreover, Wenjing Pang and colleagues reported that pancreatic cancer-secreted miR-155 implicated in the conversion from normal fibroblasts to cancer-associated fibroblast by targeting TP53INP1.^47^ Further, the function of miR-155 showed its effect on the amplification of inflammatory status in adipocytes, probably via its ability to target PPARγ,^19^ being evident that PPARγ loss attenuates the activation of hypoxia-responsive genes while increasing the levels of inflammatory genes, such as CCL5, in mature hypoxic adipocytes.^48^ Thus, it appears that miR-155 play a pivotal effect on CAC progression. However, we showed that miR-155 did not contribute to tumor-induced glycolysis in C2C12 and miR-155 inhibition could not prevent cancer-stimulated cell death. It suggested that exosomal miRNAs may have synergized effects, and other miRNA highly expressed such as miR-122 or miR-105 functioned as primary mediators observed in previous studies.^21,49^ Equally, other effectors like special protein or adrenomedullin derived from tumor exosomes may mediate the CAC change, showing that tumuor cell-released extracellular Hsp70 and Hsp90 stimulate muscle catabolism resulting in muscle wasting.^10^ Taken together, the results show that exosomes are probably exploited by cancer cells as a sort of ‘signal’ to convert the cells in CAC to satisfy the tumor growth and metastasis.

Adrenergic control of thermogenesis in muscle or fat tissue is mediated mainly by β-adrenergic receptors (β-AR), and β_3_-adrenergic receptors mainly expressed in adipocytes tissue while β_2_-adrenergic receptors primarily distributed in multiple muscle cells including skeletal muscle cells.^22,50^ Further, β_3_-Adrenergic receptor blockade was observed to ameliorate cachexia in vivo.^6^ Propranolol was found to partially reverse cancer cell–induced lipolytic activation as total β-adrenergic receptors blockade and the PPARγ activator, consisting with our findings.^14^ However, there was evidence that propranolol was not able to inhibit the lipolysis induced by tumor secretions, in contrast, catecholamines could exert a major anti-lipolytic effect by binding to α2-AR.^24,51^ Probably because propranolol was used by low dose and could fully function owing to poor selective blockade. Moreover, inflammatory effectors equally contributed to cachexia, and sulindac as anti-inflammatory drug was very effective in ameliorating the severity of cachexia and reduced UCP1 mRNA expression levels in cachectic mice.^6^ These experiments show that preventive treatments combined anti-inflammatory drugs and β_3_-AR blockade may be effective in ameliorating the severity of cancer cachexia.

We discovered that breast cancer cells-secreted exosomes triggers cancer-associated cachexia to promote metastasis by reprogramming the metabolism in adipocytes and muscle cells. Likewise, exomiR-155 may be responsible for diverse pathologic effects of tumuor on various organs either through activating their targets, or through increasing inflammatory factors. Our work suggests a new mechanism for the interaction between host cells and cancer cells mediated by exomiRNAs, and the development of therapeutics to block this interaction will be a promising strategy in cancer therapy.

### Material and methods

#### Patients

Human samples were obtained from Renmin Hospital of Wuhan University. All patients included in the study provided written informed consent, and the study was approved by the Institutional Ethics Committee of Renmin Hospital of Wuhan University. Patients did not receive financial compensation. Clinical information was obtained from pathology reports, and the characteristics of the included cases are provided in Table S1. Patients with median 5 years of follow-up were included in this study. All methods were performed in accordance with relevant guidelines and local regulations.

#### Cell culture and reagents

The human breast cancer cell lines MCF-7 and MDA-MB-231, C2C12 and HEK 293T cells were obtained from American Type Culture Collection (ATCC, Shanghai) and cultured in Dulbecco’s modified Eagle’s medium (DMEM) supplemented with 10% exosome-free fetal bovine serum (FBS, Shin Chin Industrial, SCI) and 1% penicillin–streptomycin (HyClone, Logan, UT, USA) in a humidified 37°C incubator with 5% CO_2_. 3T3-L1 preadipocytes were obtained from ATCC (Shanghai) and cultured in DMEM supplemented with 10% fetal calf serum (FCS, Gibco) and 1% penicillin–streptomycin (HyClone, Logan, UT, USA) in a humidified 37°C incubator with 5% CO_2_; these cells were differentiated as previously reported.^52^ Differentiation was confirmed by Oil Red O staining. Cytochalasin D and insulin were purchased from Sigma.

#### Coculture and migration and invasion assays

Mature 3T3-L1 and breast cancer cells were cocultured using Transwell culture plates (0.4-μm pore size; Millipore). Mature 3T3-L1 or C2C12 cells in the bottom chamber of the Transwell system were cultivated in serum-free medium containing 1% bovine serum albumin (Sigma) for 4 hours. A total of 3 × 10^5^ MCF-7 or MDA-MB-231 cells were cultivated in the top chamber in the presence or absence of mature 3T3-L1 or C2C12 cells in the bottom chamber for the indicated times. The conditioned medium (CA-CM) was collected from adipocytes cultivated with tumor cells for 3 days or C2C12 cultivated with tumor cells for 1 days. After 24 hours of coculture in the presence of normal medium or CA-CM (supplemented with 10% FBS), tumor cells were subjected to wound healing and Matrigel invasion assays.

#### Measurements of metabolites in media

The glycerol (Cayman), lactate (BioVision), pyruvate (BioVision), and FFA (BioVision) levels in media were measured using colorimetric assay kits according to the instructions from the manufacturer. The levels were normalized to protein concentration.

#### Exosome isolation and characterization

After cells were cultured with exosome-depleted serum (Shin Chin Industrial, SCI), the exosomes were purified from the conditioned medium according to the instructions.^53^ The medium was centrifuged at 500 *g* for five minutes and at 2,000 *g* for thirty minutes at 4°C to remove cellular debris and large apoptotic bodies. After centrifugation, media was added to an equal volume of a 2 × polyethylene glycol (PEG, MW 6000, Sigma, 81260) solution (final concentration, 8%). The samples were mixed thoroughly by inversion and incubated at 4°C overnight. Before the tubes were tapped occasionally and drained for five minutes to remove excess PEG, the samples were further centrifuged at maximum speed (15,000 rpm) for 1 hour at 4°C. The resulting pellets were further purified using 5% PEG and then stored in 50–100 μl of particle-free PBS (pH 7.4) at −80°C. The average yield was approximately 300 μg of exosomal protein from 5 ml of supernatant. Total RNA was extracted by using Trizol reagent (Life Technologies), followed by miRNA assessment by microarrays and RT-PCR described below. Exosomes were analyzed by electron microscopy to verify their presence, by a nanoparticle characterization system to measure their size and concentration, and by western blot to detect their proteins (TSG101, CD63 and CD81).

#### Electron microscopy

After being fixed with 2% paraformaldehyde, samples were adsorbed onto nickel formvar-carbon-coated electron microscopy grids (200 mesh), dried at room temperature, and stained with 0.4% (w/v) uranyl acetate on ice for 10 minutes. The grids were observed under a HITACHI HT7700 transmission electron microscope.

#### Nanoparticle characterization system (nanosight)

The NanoSight (Malvern Zetasizer Nano ZS-90) was used for real-time characterization and quantification of exosomes in PBS as specified by the manufacturer’s instructions.

#### Exosome uptake analysis

Exosomes derived from breast cancer cells were labeled by the cell membrane labeling agent PKH26 (Sigma-Aldrich). After being seeded in 96-well plates and allowed to differentiate, mature 3T3-L1 cells were incubated with labeled exosomes (20 μl/well) for the indicated time. Images were acquired using the Olympus FluoView FV1000.

#### Western blotting

After being washed twice with ice-cold PBS, cells were collected with SDS loading buffer and boiled for 10 minutes. The proteins were separated by SDS-PAGE, transferred to a nitrocellulose membrane, and detected with specific antibodies (Table S2).

#### RNA extraction and quantitative PCR

Gene expression was analyzed using real-time PCR. The mRNA primer sequences are provided in Table S3. The miRNA primer kits were purchased from RiboBio (Guang Zhou, China).

#### Immunohistochemistry

A cohort of 108 paraffin-embedded human breast cancer specimens was diagnosed by histopathology at Renmin Hospital of Wuhan University from 2011 to 2012. Immunohistochemistry (IHC) staining was performed, and the staining results were scored by two independent pathologists based on the proportion of positively stained tumor cells and the staining intensity. The intensity of protein expression was scored as 0 (no staining), 1 (weak staining, light brown), 2 (moderate staining, brown) and 3 (strong staining, dark brown). The protein staining score was determined using the following formula: overall score = percentage score × intensity score. Receiver operating characteristic (ROC) analysis was used to determine the optimal cut-off values for all expression levels regarding the survival rate.

#### miRNA microarrays

miRNA was isolated from exosomes with the miRNeasy Kit (Qiagen, USA), following the manufacturer’s instructions. miRNA levels were ascertained using TruSeq Small RNA Sample Prep Kits (Illumina, San Diego, CA, USA) according to the manufacturer’s instructions. ExomiRNA expression microarray data were deposited in the Gene Expression Omnibus (GEO) database (accession number: GSE109879).

#### Luciferase assays

The 3ʹ UTRs of human target genes containing predicted miRNA binding sites (gene^wt^) were cloned into the GV272 vector (GeneChem Biotechnology, Shanghai, China), and the miRNA binding sites were replaced with a 4-nt fragment to produce a mutated 3ʹ UTR (gene^mut^) in the vector. Briefly, HEK 293T cells were plated onto 12-well plates and grown to 70% confluence. The cells were cotransfected with gene^wt^ or gene^mut^, the pre-miRNA expression plasmid and pRL-SV40, which constitutively expresses Renilla luciferase as an internal control. Binding between TRAF6 and miRNA-146b was selected as the positive control.^54^ At 48 hours post-transfection, the cells were lysed, and Renilla luciferase activity was assessed by the TECAN Infiniti reader. The results are expressed as the ratio of firefly luciferase activity to Renilla luciferase activity.

#### Seahorse analyses

Cells were seeded in 24-well XF24 cell culture plates at a density of 2 × 10^4^ cells/well for 24 hours in CA-CM or AD-CM. Media were then removed, wells were washed, and the cells were incubated for 1 hour at 37°C without CO_2_ in XF modified DMEM assay medium (Seahorse Bioscience) at pH 7.4 supplemented with 1 mM glutamine, 2.5 mM glucose, 1 mM sodium pyruvate, 0.5 mM carnitine, and 1 mM palmitate complexed with 0.2 mM BSA. For glycolytic tests, the extracellular acidification rate (ECAR) was measured in the basal state (no glucose) or after the injection of 10 mM glucose, 5 μM oligomycin, and 50 mM 2DG (Sigma-Aldrich). For fatty acid oxidation (FAO) experiments, the oxygen consumption rate (OCR) was measured in the basal state (1 mM palmitate complexed with 0.2 mM BSA) or after the injection of 5 μM oligomycin, 1 μM FCCP (2-[2-[4-(trifluoromethoxy)phenyl] hydrazinylidene]-propanedinitrile), 5 μM rotenone and 5 μM antimycin A. ECAR is expressed as mpH per minute after normalization to protein content measured with a Pierce BCA Protein Assay (Thermo Fisher Scientific). OCR is expressed as pmol of O_2_ per minute after normalization to protein content.

#### Lentivirus preparation and transfection

miRNA-155 inhibitors and pre-miRNA lentiviruses were obtained from GeneChem Biotechnology (Shanghai, China). Cells were cultured at 5 × 10^5^ cells/well in 6-well plates. After being incubated for 24 hours, the cells were transfected with siRNA lentiviruses and control sequences using CON036 (GeneChem Biotechnology, China) following the manufacturer’s instructions. Cells (2 × 10^5^) were stably transfected with empty vector or with vectors carrying miRNA inhibitor or pre-miRNA using the TransIT-LT1 reagent (Mirus). Selection was carried out with puromycin (1 µg/ml, Sigma) or G418 (500 μg/ml, Sigma) in cell culture media for 48 hours after transfection. Selected clones were maintained in DMEM with 500 μg/ml G418 or 1 µg/ml puromycin. Cell lysates were collected, and RT-PCR was performed to detect miRNA expression. The sequence information is provided in Table S4.

#### Statistical analysis

All experiments were done independently at least three times. The results are presented as the mean ± SD. The relative increase in protein expression was quantified using Image J software and was normalized to control protein expression in each experiment. Data sets obtained from different experimental conditions were compared with the t-test when comparing only 2 groups. Multiple comparisons between groups were performed using the Mann–Whitney *U* test. Survival probabilities for recurrence-free survival (RFS) were estimated using the Kaplan–Meier method, and variables were compared using the log-rank test. In the bar graphs, a single asterisk (*) indicates P < 0.05.

## Abbreviations

CAC: Cancer-associated cachexia
WAT: White adipose tissue
FFAs: Free fatty acids
FATP1: Fatty acid transport protein-1
IHC: Immunohistochemistry
CytoD: cytochalasin D
FAO: Fatty acid oxidation
UCP1: Uncoupling protein-1
PPARγ: Peroxisome proliferator activated receptor γ
MYH1: Myosin heavy chain 1
CAFs: Cancer-associated fibroblasts
AMPK: AMP-activated protein kinase
PFKFB3: 6-Phosphofructo-2-kinase/fructose-2,6-biphosphatase 3
PGC-1: PPAR gamma coactivator-1
